This article has been retracted.

# Intelligent Algorithm-Based Quantitative Electroencephalography in Evaluating Cerebral Small Vessel Disease Complicated by Cognitive Impairment

**DOI:** 10.1155/2022/9398551

**Published:** 2022-01-29

**Authors:** Hengya Zhu, Jingjing Qiu, Xiaoyan Sun, Xiangyan Yang, Bin Zhang, Ying Tan

**Affiliations:** Department of Neurology, Huzhou Center Hospital, Affiliated Center Hospital of Huzhou University, No. 1558 Sanhuan North Road, Huzhou, 313000 Zhejiang, China

## Abstract

To analyze the application value of artificial intelligence model based on Visual Geometry Group- (VGG-) 16 combined with quantitative electroencephalography (QEEG) in cerebral small vessel disease (CSVD) with cognitive impairment, 72 patients with CSVD complicated by cognitive impairment were selected as the research subjects. As per *Diagnostic and Statistical Manual* (5th Edition), they were divided into the vascular dementia (VD) group of 34 cases and vascular cognitive impairment with no dementia (VCIND) group of 38 cases. The two groups were analyzed for the clinical information, neuropsychological test results, and monitoring results of QEEG based on intelligent algorithms for more than 2 hours. The accuracy rate of VGG was 84.27% and Kappa value was 0.7, while that of modified VGG (nVGG) was 88.76% and Kappa value was 0.78. The improved VGG algorithm obviously had higher accuracy. The test results found that the QEEG identified 8 normal, 19 mild, 10 moderate, and 0 severe cases in the VCIND group, while in the VD group, the corresponding numbers were 4, 13, 11, and 7; in the VCIND group, 7 cases had the normal QEEG, 11 cases had background changes, 9 cases had abnormal waves, and 11 cases had in both background changes and abnormal waves, and in the VD group, the corresponding numbers were 5, 2, 5, and 22, respectively; in the VCIND group, QEEG of 18 patients had no abnormal waves, QEEG of 11 patients had a few abnormal waves, and QEEG of 9 patients had many abnormal waves, and QEEG of 0 people had a large number of abnormal waves, and in the VD group, the corresponding numbers were 7, 6, 12, and 9. The above data were statistically different between the two groups (*P* < 0.05). Hence, QEEG based on intelligent algorithms can make a good assessment of CSVD with cognitive impairment, which had good clinical application value.

## 1. Introduction

At present, cerebral small vessel disease (CSVD) seriously endangers the lives of the elderly, and it has received increasing attention with the acceleration of aging process worldwide [1]. As with CSVD, Alzheimer's disease (AD) is a common disease in the elderly, which will lead to memory loss and decline in thinking ability. In severe cases, the patient has urinary and fecal incontinence and eventually coma, and most patients die from complicated infections [2–4]. In Northeast China, due to the special climate, the local people prefer food that is heavy in salt and sauce, which will cause the arteries and blood vessels to harden prematurely. As a result, people in this region are more likely to suffer from cerebrovascular diseases and vascular cognitive impairment (VCI) [5]. Studies have shown that CSVD is the main factor in the emergence of VCI [6]. However, the onset of CSVD is insidious and slow and it is easily ignored in the early stage. When diagnosed, it is difficult to cure. Hence, the treatment of CSVD is mainly to prevent or slow down the symptoms [7–9].

The current diagnosis of CSVD is based on neuropsychological tests, including Mini-Mental State Examination (MMSE), Montreal Cognitive Assessment (MoCA), Wechsler Adult Intelligence Scale for Republic Chinese (WAIS-RC), and Activity of Daily Living (ADL); neuroimaging examination; gait disorder assessment; and serum or cerebrospinal fluid laboratory test [10–14]. Nevertheless, such testing methods are highly subjective, and despite the strong diagnostic significance, they cannot evaluate the development trend and extent of the disease [15, 16]. The newly emerged electroencephalograph (EEG), as a laboratory neuroelectrophysiological examination, makes it more possible to diagnose CSVD, especially after the University of California, San Francisco, successfully translated brain waves into English in 2020. Compared with other diagnostic methods, EEG can directly monitor brain signals and does not require the assistance of conventional imaging. It can detect the disease before structural lesions appear, and the test can be repeated at any time [17–19]. VGG-16 algorithms have made good progress in medical diagnoses. Combining VGG-16 algorithms with EEG enables EEG to intelligently evaluate the extent of cognitive impairment caused by CSVD, that is, cerebral small vascular cognitive impairment (CSVCI), assisting medical staff in personalized diagnosis and treatment [20, 21].

In the study, 72 patients with CSVD complicated by cognitive impairment in the hospital were selected as the research subjects. According to the diagnostic criteria of the *Diagnosis and Statistics Manual of Mental Disorders* (5th Edition), they were divided into the vascular dementia (VD) group and the vascular cognitive impairment with no dementia (VCIND) group. The two groups were then compared for the clinical information, neuropsychological test results, and monitoring results based on intelligent algorithm-based quantitative electroencephalography (QEEG). The study was intended to provide a scientific basis for the diagnosis and treatment of CSVCI.

## 2. Materials and Methods

### 2.1. Research Subjects

Seventy-two patients with CSVD complicated by cognitive impairment in the hospital were selected as the research subjects. As per the *Diagnosis and Statistics Manual of Mental Disorders* (5th Edition), the patients were divided into the VD group of 34 people and VCIND group of 38 people [22]. In the VD group, there were 20 males and 14 females, with an average age of 65 ± 2.88 years. In the VCIND group, there were 24 males and 14 females, with an average age of 66 ± 3.43 years. This study was approved by the ethics committee of the hospital, and the patients and their families understood the situation of the study and signed an informed consent form.

Inclusion criteria were as follows: (I) patients who are diagnosed with CSVCI; (II) the score of the self-rating scale of depression was less than 40 points; (III) head imaging showed that there was no obvious macrovascular lesion, but lacunar cerebral infarction, cerebral microbleeds, leukoaraiosis, perivascular space enlargement, and other abnormalities were found; and (IV) the patient and their family members cooperated in the examination.

Exclusion criteria were as follows: (I) cognitive impairment caused by other central nervous system diseases; (II) cognitive impairment caused by medical system diseases; (III) patients with other serious diseases; (IV) accompanied by major mental diseases; (V) patients had other vision, hearing, and movement dysfunction and cannot cooperate in the examination; and (VI) the patients and their families were unwilling to cooperate.

### 2.2. Clinical Data of the Subjects

Clinical data of all research subjects were collected, including name, gender, history of tobacco and alcohol, history of cardiovascular and cerebrovascular diseases, and diabetes. Whether the patient was working or not and whether the head was injured were counted.

### 2.3. Cognitive Function Test

In this experiment, both the WAIS-RC scale and the MoCA scale were used to prevent omissions.

Based on the Wechsler Adult Intelligence Scale (WAIS), the WAIS-RC was adapted to conform to the humanistic and moral values with Chinese characteristics. The test includes two parts: speech and operation, a total of 12 subitems, namely, common sense, comprehension, arithmetic, similarity test, digital breadth test, vocabulary test, digital symbol test, block diagram test, picture arrangement test, graphic patchwork, and maze. The score is converted according to the attached table. A score less than 69 is considered intellectual disability, a score between 70 and 79 is considered low intelligence, a score between 80 and 89 is considered slightly normal intelligence, a score between 90 and 109 is considered normal intelligence, and a score greater than 110 is considered high intelligence.

The MoCA scale involves tests in multiple cognitive domains, and the test time is short, which is suitable for general clinical use. Compared with the WAIS-RC, it focuses on the detection of cognitive behavioral ability, including 11 tests in 8 cognitive domains: attention, concentration, execution, language, memory, thinking, vision, calculation, and space. The total score is 30 points. If the time of education is less than 12 years, 1 point will be added. A score between 26 and 30 is considered normal, and a score less than 26 points is considered cognitive dysfunction.

### 2.4. Quantitative Brain Waves Based on Intelligent Algorithms

The EEG waveforms of 100 volunteers were collected, and the EEG cognitive function database was established. 32-channel polysomnography detection system was used to monitor the numbers. According to the degree of abnormality of the EEG, it was divided into 11 types of normal EEG, lightly abnormal EEG, moderately abnormal EEG, severely abnormal EEG, the EEG with abnormal background, the EEG with abnormal waves, the EEG with abnormal background and abnormal waves, the EEG with few abnormal waves, the EEG with many abnormal waves, and the EEG with a large number of abnormal waves. The digital signal in QEEG was analyzed, and the corresponding EEG signal images were collected. Finally, 100 × 11 = 1100 pieces of data were obtained [23]. At a ratio of 3 : 7, the data was divided into verification data and experimental data. Then, the deep learning convolutional neural network is used to realize the intelligent classification of EEG images.

In this study, the Visual Geometry Group- (VGG-) 16 model (Figure 1) is used to construct the network architecture. The VGG network itself has good image classification capabilities, but in the image classification of EEG, certain improvements are required to recognize EEG dense graphics, as shown in Figure 2. The improvement is divided into 4 areas.

First, the maximum pooling layer is replaced with a convolutional layer to reduce the instability of the maximum pooling layer during the training process; second, the size of the convolution kernel of the first convolutional layer is set to 3 × 3, and the size of the rest of the convolutional kernels is 2 × 2; third, the network depth is increased by setting 6 convolutional layers in the first convolution section to process a large number of low-order features in the image; fourth, the average pooling layer replaces the fully connected layer. After the last convolutional layer outputs 512 feature maps, the average pooling layer obtains the equivalent number of outputs, and the probability is calculated by the Softmax function to reduce the complexity of the operation.

Regarding the Softmax function, there are mainly two steps; one is to convert all the prediction results into nonnegative numbers, and the other is to normalize all the results. The equations are as follows:

(1) $$\begin{array}{c} P\left(y=j\right)=\frac{\exp\left(W_{\text{j}}x\right)}{\sum_{n=1}^{N}\exp\left(W_{n}x\right)}, \end{array}$$

(2) $$\begin{array}{c} W_{j}x=\overset{d}{\underset{n=1}{\sum }}W_{jn}x_{n}=f, \end{array}$$

(3) $$\begin{array}{c} P\left(y=j\right)=\frac{\exp\left(f_{j}\right)}{\sum_{n=1}^{N}\exp\left(f_{n}\right)}=\text{softmax}{\left(f\right)}_{j}. \end{array}$$

In equations (1)–(3), *W*_j_*x* represents the output of the *j*th node, *N* represents the number of output nodes, and *P* represents the output value of the Softmax function. According to equation (2), *f*_*n*_(*j* = 1, ⋯, *n*) is calculated and substituted into equation (3).

### 2.5. Algorithm Verification

According to Figure 2, the verification data is verified. The experiment is conducted on the NVDIA GTX2080Ti GPU, Intel 2.1 GHz Xeon Silver 4110 CPU, 64 G RAM system. Th VGG improved network is constructed in the TensorFlow environment.

Then, the VGG and the improved VGG are compared for the accuracy and the Kappa value, expressed as follows:

(4) $$\begin{array}{c} \text{Accuracy}=\frac{\text{TP}}{\text{TP}+\text{FN}}=A,\\ \text{Kappa}=\frac{A‐N}{1-N}, \end{array}$$

where TP is the true-positive rate, FN is the false-negative rate, and *N* is the random classification rate.

### 2.6. Improved VGG for EEG Examination

The improved VGG was used for EEG examination on the two groups of patients. During the examination, the environment was quiet to keep the patient relaxed. Professional technicians placed electrodes according to the international 10-20 system, and the ECG and electromechanical channels were adopted at the same time. The Australian Compumedics 32-channel polysomnography system was used to monitor the patients continuously for 5 hours in both the awake and sleep periods, and the acquired data was analyzed intelligently.

### 2.7. Statistical Methods

The data was processed by SPSS19.0 version statistical software, the measurement data were expressed by the mean ± standard deviation ($\bar{x}\pm s$), and the count data were expressed by the percentage (%). One-way analysis of variance was used for pairwise comparison. The difference was statistically significant at *P* < 0.05.

## 3. Results

### 3.1. Algorithm Verification Results

Figure 3 showed the average accuracy and Kappa value of VGG and improved VGG (nVGG). It was noted from Figure 3 that the accuracy rate of VGG was 84.27% and the Kappa value was 0.7. When the improved VGG (nVGG) was used, the accuracy rate reached 88.76% and the Kappa value was 0.78. The improved VGG algorithm had a higher accuracy rate, and the difference was statistically significant (*P* < 0.05).

### 3.2. Comparison of the General Conditions of the Two Groups of Patients

The age and education level of the two groups of patients were tested by *t*-test, and the chi-square test was used for gender, history of tobacco and alcohol, history of cardiovascular and cerebrovascular diseases, diabetes, whether they had a job, and whether there was head injury. The specific results are shown in Table 1. The results showed that the differences were not statistically significant in the age, education level, gender, history of tobacco and alcohol, history of cardiovascular and cerebrovascular diseases, diabetes, whether they had a job, and whether they had head injury (*P* > 0.05).

### 3.3. Comparison of Cognitive Function between the Two Groups of Patients

Tables 2 and 3 showed the WAIS-RC score and MoCA score of the two groups of patients. It was noted from Table 2 that the two groups of patients have significant differences in 11 aspects of time, space, fast memory, concentration, mathematical calculation, language ability, visual space, and the total score under WAIS-RC, *P* < 0.05. It was noted from Table 3 that the two groups of patients had significant differences in the 8 cognitive domains of attention, concentration, execution, language, memory, thinking, vision, and calculation and space, as well as the total score, *P* < 0.01.

### 3.4. Recognition and Classification Results of the Improved VGG for the Two Groups of Patients

Figure 4 showed the EEG of patients in the VD group identified by modified VGG. The slow wave rhythm originated from the left temporal part gradually evolved into sharp wave rhythm. According to Figure 5, there were 12 normal images, 32 mildly abnormal images, 21 moderately abnormal images, and 7 severely abnormal images. Specifically, they were 8, 19, 10, and 0 for VCIND; for VD, they were 4, 13, 11, and 7, respectively. There were statistical differences between the above two groups (*P* < 0.05). As shown in Figure 6, there were 12 cases of normal images, 13 cases of only background changes, 14 cases of abnormal waves only, and 33 cases of both the background and wave changes. Specifically, they were 7, 11, 9, and 11 for VCIND; for VD, they were 5, 2, 5, and 22, respectively. There were statistical differences between the above two groups (*P* < 0.05). According to Figure 7, there were 25 cases without abnormal waves, 17 cases with a few abnormal waves, 21 cases with many abnormal waves, and 9 cases with a large number of abnormal waves. Specifically, for VCIND, they were 18, 11, 9, and 0; for VD, they were 7, 6, 12, and 9 cases, respectively. There were statistical differences between the above two groups (*P* < 0.05).

### 3.5. Relationship between EEG Classification and Cognitive Function

The changes in the EEG corresponded to the differences in the WAIS-RC score and the MoCA score, as shown in Table 4. According to Table 4, the WAIS-RC and MoCA scores were statistically different between the 4 groups (*P* < 0.05).

## 4. Discussion

CSVD refers to the changes in the cognitive function, neuroimaging, and neuropathology arising from diseases of small arteries, venules, capillaries, and small perforating arteries with a diameter of 40-200 *μ*m, mainly the CSVCI. CSVCI mainly manifests as the impairment of daily basic abilities, such as self-care ability, cognitive ability, execution ability, and thinking ability, especially the execution ability. It is currently believed that this is related to damage to the cortex-subcortical fibrous circuit. The impairment of the hippocampus-medial temporal lobe-subcortical function will cause the decline in memory function, but the degree is not as obvious as Alzheimer's disease.

The diagnosis of CSVCI is mainly based on the neuropsychological evaluation, including WAIS-RC, MoCA, ADL, MMSE, and other evaluation forms. The WAIS-RC is currently the most widely used clinical intelligence assessment scale. It has a wide detection range and strong sensitivity and specificity for intelligence detection but is not sensitive to cognitive impairment. MoCA is an important scale used to quickly screen patients with mild cognitive impairment [17]. Combining the two can guarantee a complete screening of patients with cognitive impairment.

However, all of the above scales have limitations in judging the development and severity of the disease. EEG is a common electrophysiological examination method and highly sensitive to brain cell function and can be used for the prediction, identification, diagnosis, evaluation, and differentiation of symptoms such as dementia. With the rise of artificial intelligence, the intelligent algorithms can help to improve the accuracy of EEG.

In the study, patients with CSVCI were selected as the research subjects and divided into the VCIND group and VD group. First, the clinical data of patients between the two groups were analyzed, and it was determined that *P* > 0.05, indicating that the difference was not statistically significant. Then, WAIS-RC and MoCA tests were performed. At the same time, the improved VGG algorithm was used for training to improve its recognition ability and accuracy. The verification experiment showed that the accuracy of the improved VGG after was 88.76%, higher than 84.27% before the improvement. It proved that the improved algorithm can elevate the recognition ability of EGG. Next, the two groups of patients were monitored for 5 hours continuously. The EGG can be trained to recognize the required image data. This study found that the abnormal rate of EEG of CSVCI was 83.4%. Specifically, the abnormal rate in the VCIND group was 78.9% and the abnormal rate in the VD group was 88.2%. Of the CSVCI patients, 44.4% had mild abnormalities, 29.2% of moderate abnormalities, and 9.7% of severe abnormalities. In the VCIND group, the corresponding percentages were 21.1%, 50%, and 0%; in contrast, they were 38.2%, 32.4%, and 20.6% in the VD group. Subsequently, the results were compared with the evaluation results of WAIS-RC and MoCA scales, and it was found that in terms of VCIND and VD identification, both the two methods performed well. However, the VCIND group was mainly the mild and moderate abnormalities, and the degree of abnormality increased with the development of the disease. Experiments confirmed that QEEG based on intelligent algorithms was sensitive to VCIND and that not only can it identify VCIND and VD, but also can reflect the development of the disease complicated by cognitive impairment. According to the study of Liedorp et al. [24] on the EEG of 1116 patients with cognitive impairment, the EEG with only the focal abnormalities can diagnose mild cognitive impairment; the EEG with only diffuse abnormalities can diagnose Alzheimer's disease; and the EEG with both focal and diffuse abnormalities supported the diagnosis of vascular dementia, dementia with Lewy bodies, and Alzheimer's disease.

This study found that the normal EEG rate of patients with CSVCI was 16.7%, the EEG with only background changes accounted for 18.1%, the EEG with abnormal waves accounted for 19.4%, and the EEG with both abnormal background and abnormal waves accounted for 45.8%. Specifically, the normal rate in the VCIND group was 21.1%, and the normal rate in the VD group was 11.8%.In the VCIND group, the background changes only accounted for 26.3%, the abnormal waves only accounted for 23.7%, and both the background changes and the abnormal wave accounted for 28.9%; in contrast, they were 8.8%, 14.7%, and 64.7% in the VD group. The analysis of the abnormal waves found that 23.6% had a few abnormal waves, 29.2% had many abnormal waves, and 12.5% had a large number of abnormal waves. In the VCIND group, 28.9% had a few abnormal waves, 23.7% had many abnormal waves, and 0% had a large number of abnormal waves; in contrast, they were 17.6%, 35.3%, and 26.5% in the VD group, and all abnormal waves were unilateral or bilateral frontal or (and) temporal lobe focal abnormal waves, mainly the sharp waves, spike waves, sharp waves, and spike waves. This showed that when the CSVCI does not develop into moderate to severe dementia, the EEG mainly shows the background change. When the cognitive function impairment is further aggravated, the EEG shows background changes as well as the abnormal waves, providing a scientific basis for judging the course of cognitive impairment.

## 5. Conclusion

In the study, the intelligent algorithm was incorporated into the EEG to improve its recognition and cognitive ability of CSVD with cognitive impairment. Then, the EEG diagnostic results were compared with the results of WAIS-RC and MoCA results. It was found that the EEG can not only identify VCIND and VD but also reflect the degree of development of VCIND, providing a more accurate and effective method for the clinical diagnosis of CSVD with cognitive impairment. In the meanwhile, it also provides test ideas for the diagnosis and treatment of various cognitive disorders in the future. However, some limitations in the study should be noted. The sample size is small, which will reduce the power of the study. In the follow-up, an expanded sample size is necessary to strengthen the findings of the study. It is believed that this research can provide ideas and experimental support for the development of diagnostic techniques for cognitive impairment in the future.

## Figures and Tables

**Figure 1:** VGG-16 network model.

**Figure 2:** Improved VGG network model.

**Figure 3:** The effect of VGG and nVGG on the results. Note: ∗ indicated that the difference was statistically significant compared with the improved nVGG algorithm (*P* < 0.05).

**Figure 4:** Improved VGG identifying EEG of patients in the VD group.

**Figure 5:** EEG classification of the two groups of patients: (a) the CSVCI group; (b) the VCIND group; (c) the VD group.

**Figure 6:** The overall changes of the EEG of the two groups of patients: (a) the CSVCI group; (b) the VCIND group; (c) the VD group.

**Figure 7:** The distribution of abnormal EEG waves in the two groups of patients: (a) the CSVCI group; (b) the VCIND group; (c) the VD group.

**Table 1:** Comparison of the general conditions of the two groups of patients.

	VCIND	VD	*P*
Age (year)	66 ± 3.43	65 ± 2.88	0.236
Degree of education (year)	9.89 ± 2.782	10.03 ± 2.746	0.302
Sex (man/woman)	24/14	20/14	0.427
Cardiovascular and cerebrovascular diseases (no/yes)	34/4	32/2	0.886
Head injuries (no/yes)	2/36	1/33	0.892
Diabetes (no/yes)	21/17	20/14	0.942
Job (no/yes)	19/19	21/13	0.431
Liquor & tobacco (no/yes)	23/11	22/12	0.307

**Table 2:** The score of each item of WAIS-RC (mean ± standard deviation).

WAIS-RC	VCIND	VD	*P*
Total points	87.06 ± 12.109	76.87 ± 13.892^∗^	≤0.001
Information	6.52 ± 0.873	4.89 ± 2.145^∗^	≤0.001
Similarities	6.67 ± 0.429	4.29 ± 1.333^∗^	0.001
Vocabulary	6.17 ± 1.008	4.01 ± 2.04^∗^	≤0.001
Arithmetic	6.08 ± 1.112	4.11 ± 2.01^∗^	0.002
Comprehension	5.41 ± 0.802	4.93 ± 1.364^∗^	≤0.001
Digit span	5.39 ± 1.371	4.62 ± 0.979^∗^	≤0.001
Picture completion	4.62 ± 0.882	4.15 ± 0.791^∗^	≤0.001
Picture arrangement	5.29 ± 1.021	4.82 ± 0.892^∗^	≤0.001
Block design	6.01 ± 1.028	5.06 ± 1.031^∗^	≤0.001
Object assembly	8.24 ± 0.683	8.11 ± 1.262^∗^	≤0.001
Maze	3.67 ± 0.551	3.01 ± 1.002^∗^	≤0.001
Digit symbol	3.47 ± 0.573	2.07 ± 0.491^∗^	0.018

∗ indicated that the difference was statistically significant compared with the VCIND group.

**Table 3:** The score of each item in the MoCA scale (mean ± standard deviation).

MoCA	VCIND	VD	*P*
Total points	21.87 ± 3.691	13.16 ± 2.892^∗^	≤0.001
Attention	2.98 ± 1.201	1.61 ± 1.301^∗^	0.035
Execution	2.36 ± 1.106	1.59 ± 2.011^∗^	0.001
Memory	2.19 ± 0.821	1.68 ± 1.012^∗^	≤0.001
Thinking	0.69 ± 0.701	0.38 ± 0.622^∗^	0.021
Vision	2.81 ± 0.891	2.12 ± 0.677^∗^	≤0.001
Language	1.89 ± 0.932	1.66 ± 0.791^∗^	≤0.001
Computation	2.01 ± 0.712	1.85 ± 0.641^∗^	≤0.001
Space	5.33 ± 1.006	2.88 ± 1.376^∗^	≤0.001

∗ indicated that the difference was statistically significant compared with the VCIND group.

**Table 4:** Relationship between EEG classification and WAIS-RC and MoCA scores (mean ± standard deviation, scores).

	Normal	Mild	Moderate	Severe	*P*
WAIS-RC	21.27 ± 3.915	21.98 ± 6.012	19.86 ± 5.612	13.37 ± 4.602	0.006
MoCA	17.54 ± 5.234	16.84 ± 4.995	15.39 ± 5.027	8.15 ± 1.374	0.002

## Data Availability

The data used to support the findings of this study are available from the corresponding author upon request.
